The article "Effect of Respiration Training-Assisted Western Medicine Therapy on Activity Tolerance, Pulmonary Function, and Quality of Life of Chronic Obstructive Pulmonary Disease Patients in the Stable Phase" was retracted in 2023. Reason: concerns about the peer review.

# Effect of Respiration Training-Assisted Western Medicine Therapy on Activity Tolerance, Pulmonary Function, and Quality of Life of Chronic Obstructive Pulmonary Disease Patients in the Stable Phase

**DOI:** 10.1155/2022/9427602

**Published:** 2022-03-30

**Authors:** Yaqi Tong, Jia Cui, Di Chai

**Affiliations:** Department of Respiratory and Critical Care Medicine, Beijing Hospital, Beijing 100730, China

## Abstract

**Objective:**

To explore the effect of respiration training-assisted western medicine therapy on activity tolerance, pulmonary function, and quality of life (QOL) of chronic obstructive pulmonary disease (COPD) patients in the stable phase.

**Methods:**

The medical data of 90 COPD patients in the stable phase treated in the respiratory medicine of our hospital (November 2020–November 2021) were chosen for the retrospective analysis, and the patients were split into group A (*n* = 45, respiration training-assisted western medicine therapy) and group B (*n* = 45, western medicine therapy) according to the clinical reception order, so as to record and compare the activity tolerance, lung function, and QOL between the groups after intervention.

**Results:**

Compared with group B after intervention, group A showed greatly longer mean 6-min walking distance, significantly lower St. George's Respiratory Questionnaire (SGRQ) score, significantly higher specific airway conductance (sGAW) and level values of various lung function indicators, and significantly lower level values of airway resistance (RAW) and specific airway resistance (sRAW) (*p* all<0.001); the total effective rate was significantly higher in group A (*p* < 0.05).

**Conclusion:**

Respiration training-assisted western medicine therapy is a dependable way to improve the activity tolerance of COPD patients in the stable phase, and such strategy largely improves patients' lung function and QOL. Deeper studies will be helpful to establish a preferable solution for such patients.

## 1. Introduction

Chronic obstructive pulmonary disease, abbreviated as COPD, is a clinically common respiratory disease with high morbidity and mortality [1]. Its pathogenic factors are smoking, air pollution, inhalation of dust and harmful gases, and respiratory tract infection. The disease is clinically distinguished by persistent respiratory symptoms and airflow limitation [2], severely affecting patients' life safety and at the same time causing a heavy economic burden on patients and their families. With the continuously deepened clinical research in recent years, attention has been paid to respiratory training in clinical work for patients with stable COPD [3, 4]. Recently, much attention has been paid to respiratory training, which has achieved the goal of improving lung function of patients through exercises such as glottic vocalization training and breathing exercise. Some scholars believe [5] that performing respiratory training for COPD patients is able to effectively improve their respiratory function, thus resulting in improved pulmonary function, and this training modality has been demonstrated in patients with cancer complicated by stroke, stroke hemiparesis, and chronic rotator cuff injury [6–8]. Western medicine can effectively improve many discomfort symptoms in patients, and it plays an important role in anti-inflammation and improving diaphragm function. Furthermore, the combination of *β*_2_ receptor agonists, glucocorticoids, and other western medicines can also expand the airways of patients, which can greatly alleviate their symptoms such as asthma, breathlessness, and shortness of breath, but long-term medication easily causes immune function reduction, airway fungal infection, etc., so other supplementary rehabilitation treatments are needed [9]. Currently, there are no studies confirming the effect of respiratory training-assisted western medicine therapy on activity tolerance, lung function, and quality of life (QOL) of stable COPD patients. This study further analyzed the efficacy of the combined therapy on stable COPD patients, in the hope of providing guidance for the treatment of such patients, with the results reported as follows.

## 2. Materials and Methods

### 2.1. General Data

Ninety COPD patients in the stable phase treated in the respiratory medicine of our hospital (November 2020–November 2021) were chosen as the subjects and randomly split into groups A and B based on the clinic reception sequence. After admission, all patients received relevant examinations. The study met the World Medical Association Declaration of Helsinki (2013) [10].

### 2.2. Inclusion and Exclusion Criteria

Inclusion criteria were as follows: ① the patients who met the diagnostic criteria for COPD proposed in Global Initiative for Chronic Obstructive Lung Disease (GOLD) [11] in 2018 were in the stable phase at the time of enrollment (i.e., appearance of minor chest distress, gasping, cough, anorexia) and had a stable condition for nearly 4 weeks; ② the patients were conscious and could go a long with relevant examinations such as cardiopulmonary examination; and ③ the patients presented no allergic reactions to the drugs used herein.

Exclusion criteria were as follows: ① the patients were complicated with severe heart, kidney, liver, muscle, and other systemic diseases; ② the patients suffered from airflow limitation caused by bronchitis, bronchiectasis, bronchial asthma, pulmonary *tuberculosis*, etc., and ③ the patients were unconscious or had poorer compliance.

### 2.3. Methods

Patients in group B received western medicine therapy, and the antibiotic was selected according to the susceptibility results and medical history (with or without *Pseudomonas aeruginosa* infection risk); 0.5 mg of compound ipratropium bromide solution (manufacturer: Laboratoire Unither; registration number: H20150158; specification: (2 ml: 250 *μ*g) ^∗^ 10 bottles) was administered via oxygen drive atomization, 3 times a day; 1 mg of budesonide solution (manufacturer: AstraZeneca Pty Ltd.; approval number: H20140475); specification: 1 mg: 2 ml ^∗^ 5 bottles) was administered via oxygen drive atomization, 2 times a day; and 30 mg of ambroxol hydrochloride injection (manufacturer: TIPR Pharmaceutical Responsible Co., Ltd.; NMPA approval no. H20051604; specification: 4 ml: 30 mg) was administered via intravenous injection, 2 times a day; other symptomatic supportive care was given for 14 d.

Patients in group A received the respiratory training-assisted western medicine therapy (the methods of applying western medicines were the same as above). The respiratory training mainly included 4 parts. ① Breathing exercise: patients clinched their hands, slowly raised, and put down the hands rhythmically, breathed in when raising, and breathed out when putting down; fully relaxed their scapula, and took a deep breath through the nose, and then did pursed-lip breathing; ② with exercises such as blowing out candles, blowing balloons, blowing a whistle, blowing bubbles, and playing the flute, patients could deepen the amplitude of respiration and increase the ventilation volume, so as to discharge alveolar residual gas, improve and enhance the pulmonary function; ③ glottis voice training: the patients were instructed to breathe deeply through the nose—hold the breath—and push the palm to make vowel sounds of “a”, “u”, and “e”, 5–10 times each, one set of tones were trained 3–5 times in a row, and sounder, breathing trainer, and other tools could also be applied to help them in producing sound; ④ abdominal breathing: the patients were in the supine position with knees bent and were instructed to inhale through the nose and exhale through the mouth. At the end of expiration, the physician put a hand on the patients' upper abdomen and slightly applied pressure along the direction of the upper diaphragm, and the patient exhaled under such pressure.

### 2.4. Efficacy Evaluation Indicators

#### 2.4.1. Activity Tolerance

After intervention, all patients carried out the 6-minute walk test. By means of walking, the distance that a patient can walk at the fastest speed they can tolerate within 6 min was measured. This experiment is a supplement to cardiopulmonary exercise testing and a guidance for the development of cardiac rehabilitation in primary hospitals, which can evaluate the severity of the disease and prognosis of patients. The longer distance indicated better activity tolerance.

#### 2.4.2. Respiratory Function

The airway resistance (RAW), specific airway resistance (sRAW), and specific airway conductance (sGAW) were measured with the volume scanner (specification: Astograph Jupiter-21; manufacturer: CHEST).

#### 2.4.3. Lung Function

Before testing, the patients rinsed and cleaned their mouth to avoid respiratory infectious disease or bad breath. In a comfortable sitting position, the patients were guided to do the deep breathing exercise, that is, inhaling hard and then exhaling with the maximum speed and effort, and after repeated training, the measurement was conducted. First, the patients' nose was clipped with a nose clip, and then, a disposable mouth pipette connected to the spirometer (purchased from Biobase Biodustry (Shandong) Co., Ltd.; model: FGC-A+) was placed in the subjects' mouth to do deep breathing and measure FEV1, PEF, and FEV1/FVC. After measurement, the patients stayed for 20-min observation and could leave in case of no discomfort symptoms.

#### 2.4.4. Efficacy Evaluation

The curative effect of the patients was assessed with the mMRC (modified Medical Research Council) Dyspnea Scale [12]. The scale divided the degree of activity, that is, the patients experienced shortness of breath, into 4 grades (grade 0, dyspnea only with strenuous exercise; grade 1, dyspnea when walking on flat ground or walking up a slight hill; grade 2, walks slower than people of the same age because of dyspnea or has to stop for breath when walking at own pace; grade 3, stops for breath after walking 100 m or after a few minutes; grade 4, too dyspneic to leave the house or breathless when dressing). And compared with the scores of pretherapy, a 2-point increase in the mMRC score of the patients was considered as markedly effective, a 1-point increase was considered as effective, and failure to increase was considered as ineffective.

#### 2.4.5. QOL Evaluation

Patients' QOL was evaluated by St. George's Respiratory Questionnaire (SGRQ) [13], which, by adopting the method of weighting mean, was scored according to the weighting, with less scores indicating a smaller impact on life. Within the range of 0–100 points, 0 point meant no impact at all, and 100 points meant the extreme impact on life.

### 2.5. Statistical Methods

In this study, the data were processed with the professional statistics software SPSS26.0, the picture drawing software was GraphPad Prism 7 (GraphPad Software, San Diego, USA), the enumeration data were examined by X^2^ test and expressed by (n(%)), the measurement data were examined by *t*-test and expressed by mean ± SD, and differences were considered statistically significant at *p* < 0.05.

## 3. Results

### 3.1. General Data

Table 1 shows that no significant between-group differences in the clinical data such as gender ratio, severity of illness, family economic situation, and place of residence were observed (*p* > 0.05).

### 3.2. Activity Tolerance

Figure 1 shows that group A obtained a significantly longer posttreatment mean 6-min walking distance of patients than group B (*P* < 0.001).

### 3.3. Respiratory Function

Table 2 shows that after treatment, group A obtained significantly higher sGAW level values and significantly lower RAW and sRAW level values than group B (P all<0.001).

### 3.4. Lung Function

Table 3 shows that group A obtained various posttreatment lung function indicators than group B (*P* < 0.001).

### 3.5. Clinical Efficacy

Table 4 shows that group A achieved a significantly higher total effective rate than group B (*p* < 0.05).

### 3.6. QOL

Figure 2 shows that group A acquired a significantly lower posttreatment SGRQ scores than group B (*p* < 0.001).

## 4. Discussion

COPD is a chronic respiratory disease caused by long-term exposure to toxic particles or harmful gases that leads to pathological changes throughout the respiratory system, including the airways, lung parenchyma, pulmonary alveolar, and pulmonary vasculature [5]. A clinical survey in China has shown [14,15] that COPD is prevalent in people over 40 years old, and the disease may rank 3rd for fatal diseases and 5th for the economic burden of diseases in the world. COPD mortality is increasing year by year, the economic burden is aggravating, and its incidence population tends to become younger [16]. The pathogenic factors of COPD include smoking, inhalation of dust, air pollution, repeated respiratory tract infection, and heredity. Therefore, it has become an important public health issue to initiate early interventions for COPD patients to control the development of their condition, reduce mortality, and relieve the economic burden on the diseased group.

The occurrence of COPD is related to the chronic inflammation of the airways and lung parenchyma caused by harmful gases and particles, which can also further develop to airway remodeling and then aggravate the hypoxic state in the body and pulmonary ventilatory dysfunction [17]. Because of the progressive decline in lung function, even patients in the stable phase of the disease experience activity limitation and reduced QOL. Currently, one of the most significant treatments for stable COPD in western medicine is antibiotic treatment, but using antibiotics for a long time may lead to many side effects such as osteoporosis, hoarseness, and oral flora derangement, which may cause secondary harm to them [18, 19]. Clinical studies have found that most COPD patients show declined respiratory muscle strength and endurance, and by implementing respiratory training, the respiratory muscle strength and endurance of patients can be enhanced to a certain extent. Breathing exercise effectively increases the patients' breathing strength and greatly elevates the breathing time and the gas exchange frequency, and abdominal breathing elevates the patients' exercise capacity, respiratory muscle strength, and endurance, which are good for promoting the recovery of impaired respiratory function and sputum excretion, thereby greatly reducing the frequency of disease attacks and improving the QOL [20]. The rehabilitation training for stable COPD was applied earlier in European and American countries, but it is still in the initial stage in China. Respiratory training can improve patients' systolic and diastolic function of respiratory muscles and then increase alveolar ventilation and improve lung function [21]. Drawing on previous clinical treatment experience, this study was designed to offer new ideas for the improvement of lung function in patients with stable COPD by conducting clinical controlled studies. The study results showed that group A obtained significantly longer posttreatment 6-min walking distance than group B (*p* < 0.001), demonstrating that implementing respiratory training based on western medicine therapy can greatly promote the activity tolerance of COPD patients, and the reason may be that respiratory training can play the role of delaying the expiratory flow rate, increasing the gas exchange, and elevating the blood partial pressure of oxygen and the oxygen saturation, which effectively reduces the partial pressure of carbon dioxide and the respiratory rate of the patients' arteries and greatly improves the clinical symptoms such as shortness of breath, thereby fundamentally increasing the respiratory rate [22]. In terms of the improvement of lung function, group A obtained significantly higher various posttreatment lung function indicators than group B (*p* < 0.001), implying that the combined intervention measures can obviously enhance the lung function of stable COPD patients, and the reason may be that respiratory training is helpful to enhance the endobronchial pressure, enlarge the inner diameter of bronchus, prevent premature bronchial occlusion, increase the time of gas exchange in lungs, reduce carbon dioxide retention, and improve lung function, as demonstrated in chronic refractory heart failure with sleep disturbances [23]. As for the QOL, this study applied SGRQ scoring to patients in the two groups after intervention, and the result showed that group A obtained a significantly lower SGRQ score than group B (*p* < 0.001), which may be due to the fact that respiratory training-assisted western medicine therapy can obviously improve the lung function and activity tolerance, increase the effective ventilation of the pulmonary alveoli, reduce carbon dioxide retention, and increase exercise tolerance of stable COPD patients, thereby promoting their QOL [24].

The shortcomings of the study included lacking a comprehensive evaluation of muscle strength and endurance, short follow-up observation time, and failure to carry out the long-term follow-up and observe the long-term outcomes of the patients. Therefore, further studies and clinical tests are required.

## Figures and Tables

**Figure 1:** Between-group difference in patients' 6-min walking distances (mean ± SD). *Note.* The horizontal axis denoted groups A and B, and the vertical axis denoted the 6-min walking distance (m); the mean 6-min walking distances of groups A and B were, respectively, (369.32 ± 14.22) and (284.24 ± 18.55); and ^*∗*^ indicated a significant between-group difference in the posttreatment mean 6-min walking distances (*t* = 24.418, *p* < 0.001).

**Figure 2:** SGRQ scores (mean ± SD). *Note.* The horizontal axis denoted groups A and B, and the vertical axis denoted the SGRQ score (points); the SGRQ scores of groups A and B were, respectively, (28.87 ± 4.05) and (35.47 ± 4.24); and ^*∗*^ indicated a significant between-group difference in SGRQ scores (*t* = 7.551, *p* < 0.001).

**Table 1:** Between-group comparison of general data (*n* = 45).

Item	Group A	Group B	*X* ^2^/*t*	*p*
Gender			0.178	0.673
Male/female	23/22	21/24		
Mean age (mean ± SD, years)	61.98 ± 4.53	62.13 ± 3.78	0.171	0.865
BMI (mean ± SD, kg/m^2^)	22.06 ± 1.35	22.40 ± 1.32	1.208	0.230
Mean course of disease (mean ± SD, years)	6.56 ± 1.57	6.76 ± 1.73	0.574	0.567
Severity of illness				
Mild	12 (26.67%)	13 (28.89%)	0.055	0.814
Moderate	17 (37.78%)	19 (42.22%)	0.185	0.667
Severe	16 (35.56%)	13 (30.95%)	0.458	0.499
Family economic situation			0.045	0.832
≥3,000 yuan (month·person)	25 (55.56%)	24 (53.33%)		
<3,000 yuan (month·person)	20 (44.44%)	21 (46.67%)		
Place of residence (n(%))			0.182	0.670
Urban area	25 (55.56%)	27 (60.00%)		
Rural area	20 (44.44%)	18 (40.00%)		
Educational degree (n(%))				
Junior college and above	4 (8.89%)	6 (13.33%)	0.450	0.502
Senior high school	9 (20.00%)	10 (22.22%)	0.068	0.796
Junior high school and below	32 (71.11%)	29 (69.05%)	0.458	0.499

**Table 2:** Between-group differences in respiratory function (mean ± SD).

Group	*n*	sGAW (%)	RAW (L/s)	sRAW (%)
A	45	64.16 ± 2.68	128.43 ± 3.85	128.91 ± 9.50
B	45	56.24 ± 1.83	167.41 ± 4.29	142.66 ± 7.56
t		16.372	45.363	7.597
P		<0.001	<0.001	<0.001

**Table 3:** Between-group differences in lung function (mean ± SD).

Group	*n*	FEV1 (L)	PEF (L/S)	FEV1/FVC (%)
A	45	1.99 ± 0.14	7.82 ± 0.27	73.59 ± 7.36
B	45	1.58 ± 0.26	5.05 ± 0.14	60.56 ± 4.50
*t*		9.314	61.096	10.132
*p*		<0.001	<0.001	<0.001

**Table 4:** Between-group difference in clinical efficacy (n(%)).

Group	*n*	Markedly effective	Effective	Ineffective	Total effective rate
A	45	18 (40.00)	25 (55.56)	2 (4.44)	95.56% (43/45)
B	45	10 (22.22)	27 (60.00)	8 (17.78)	82.22% (37/45)
*X* ^2^					4.050
*p*					<0.05

## Data Availability

The data used to support the findings of this study are available on reasonable request from the corresponding author.
